The article "The Construction of Basketball Training System Based on Motion Capture Technology" was retracted in 2023. Reasons: signs of a paper mill; suspected computer-generated content; unreliable results or conclusions; lack of ethics approval or compliance.

# The Construction of Basketball Training System Based on Motion Capture Technology

**DOI:** 10.1155/2021/2481686

**Published:** 2021-09-15

**Authors:** Shangqi Nie, Yuanqing Li, Biao Ma, Yufeng Zhang, Jeho Song

**Affiliations:** ^1^School of Physical Education, Huanghuai University, Zhumadian, China; ^2^Department of Sports Science, Wonkwang University, Iksan-si, Republic of Korea

## Abstract

Motion capture is a cross-cutting application field developed in recent years, which comprises electronics, communications, control, computer graphics, ergonomics, navigation, and other disciplines. The accurate application of basketball technical movements in the basketball game is very important. Therefore, it is of great significance to capture and standardize athletes' movements and improve their training. Unfortunately, there are numerous issues in traditional classroom teaching that largely helps to train the athletes. To solve the issues of traditional basketball classroom teaching, a virtual simulation system for students' sports training is designed in this paper. Firstly, the information of basketball dribbling movement is captured and simulated in three dimensions. Secondly, we compare it with the standard database to judge the irregularities of athletes' movements, and carry out digital processing on athletes' movements and skill improvements statistics in combination with system functions. Thirdly, we set up a gradual training cycle. Finally, the Kinect-based capture technology is adopted to obtain the activity information of different joints of the human body. Through processing the motion data, relevant motion analysis data are fed to the established motion model, to realize the comparative analysis of motion pictures. In our experiments, we observed better training of the physical education.

## 1. Introduction

Basketball is a collective sport that puts the ball into the opponent's basket to score points and prevents the opponent from getting the ball and scoring points under specific rules. Compared with other ball games, basketball has many skills, various tactical forms, and strong skills of players, which also reflects the characteristics of individual combat and cooperation [1]. With the national requirements for quality education, more and more colleges and universities begin to use information technology to realize the auxiliary teaching of physical education. At the same time, with the aid of the development of simulation system, students' learning of the physical education and professional technology is promoted. The 13th Five-Year Plan for education informatization emphasizes deepening the application of technology, integrating technological innovation, realizing the modernization of education through education informatization, and building a networked, digital, personalized, and lifelong education system. Moreover, its purpose is to actively apply new technologies to transform the traditional teaching mode [2]. Using multimedia database system can provide more vivid learning materials for students, thus improving students' interest in learning. Using advanced multimedia system can also help analyze multiple videos in real time. There are many basketball fans in our countries, but there is a shortage of basketball training, especially in the training methods, which are somewhat different from those of developed countries [3]. Basketball trains its own operation skills by imitating specific movements. Basketball players often imitate, observe, and correct movements. Therefore, physical training should strengthen the practice of vision and hearing. Currently, basketball teaching learns basketball skills through observing teachers' demonstration movements.

The motion capture method, which is based on inertial sensing, uses microelectromechanical or electromagnetic elements and arranges them at multiple joint points of the human body. Furthermore, it obtains motion capture results by fusing and calculating inertial data of various limb parts in the motion process [4]. The recognition technology of image analysis mainly carries out the recognition of human body posture by collecting information such as videos and images. Therefore, monitoring equipment such as cameras and sensors needs to be placed in advance in the detection environment to carry out data collection. The image analysis technology has been applied to the recognition of human body posture earlier [5]. In basketball training, the training process can be combined with the computer basketball training system, and personalized recommendations can be made according to the individual characteristics of the players. This gives full play to the individual advantages of the basketball players and improves the sports efficiency of the players. The motion capture method based on inertial sensing does not suffer from occlusion, has no light influence, can be used indoors and outdoors, and is easy to realize all-weather and unrestricted motion capture [6, 7]. However, it also has certain defects. For example, the number, layout, performance, and attitude calculation algorithms of sensors all affect the accuracy, dynamic characteristics, and stability of the motion capture. Therefore, there exist significant research gaps that should be investigated to improve the training process of the athletes. In this paper, we utilize the motion capture technology for improving the basketball teaching. Following are the major contributions of the research conducted in this paper:

1. To effectively integrate motion capture and basketball teaching.
2. To design and develop high-quality innovative teaching and training resources.
3. To provide new ideas for the design and development of basketball teaching and training.
4. To contribute to the promotion of physical education reform.

The structure of the remaining part of this paper is as follows. An overview of the related work, in terms of games and motion capture technology, is given in Section 2. In Section 3, we briefly describe the motion capture technology and its application in games.  Section 4 describes the details of the research methodology. In Section 5, we discuss the results of our work.  Section 6 presents the analysis and discussion of the findings of our study. Finally, Section 7 concludes this paper and provides directions for further research and investigation.

## 2. Related Work

In the basketball industry, ornamental consumption and equipment consumption are the two pillars of the industry profits. With the development of science and technology, the concept of intelligence has gradually penetrated all aspects of the modern market. Combining and integrating intelligence with sports products and creating intelligent sports training equipment are the mainstream elements in the current markets [8, 9]. At present, motion capture is mainly divided into two sections according to the development trend: (i) optical motion capture method and (ii) inertial sensing motion capture method. The optical-based motion capture method requires setting an optical mark on the captured object, in advance, and then capturing the spatial position of a specific light spot on the object through a high-speed camera to complete the task of motion capture [10]. Due to the particularity of physical education, there are some problems in the application of teaching and training in physical education, such as difficulty in recording and shooting, and insufficient application ability of computer technology in the process of video editing and production by physical education teachers [11].

Xia et al. [12] have conducted relevant research on key frame extraction of human motion capture data based on joint kernel sparse representation. Boukhayma and Boyer [13] proposed the synthesis theory of surface motion capture animation. Wang et al. [14] studied the proposition of outdoor unlabeled motion capture with handheld cameras. Based on the analysis of relevant documents and teaching competition works in national universities, it is found that the current basketball teaching and training still cannot break through the shackles of traditional demonstration teaching methods in teaching design [15]. In addition, it is difficult to avoid wrong movements and possible injuries to athletes' muscles, soft tissues, and bones through scientific observation during the training. These issues will further affect the normal training and even shorten the athletes' sports life [16, 17]. Basketball motion capture system has high image feature extraction ability, which can be used in the design of picking robot vision system to effectively improve the system's target recognition ability and improve the level of automated operations.

## 3. Motion Capture Technology

The goal of this paper is to realize real-time tracking of real human motion by 3D model through inertial sensing method. Human motion capture based on motion sensing is to place sensors at key nodes of human body to collect posture information in the process of human motion in real time and calculate characteristic parameters of human motion process through data fusion and calculation. The main function of user identification is to detect the identity of visitors and grant them different rights according to their identities. User identification is a must for all systems and is related to the safety and operation of the system. The system can capture the motion of the game video frame in real time and count the technical motion data from the motion features, thus obtaining the multimedia data support of the basketball technical motion [18]. Under different capture environments, the marker balls reflecting near-infrared rays are collected and recorded by setting the focal length, aperture, gray scale, and angle of the camera. Moreover, the motion track of the key points at the positions where the marker balls are located is accurately captured. To achieve realistic rendering effect, the athlete model established by the system has accurate size and structure for observation [19]. The working principle of the hardware is to continuously emit infrared rays into the whole space through an infrared emitter and encode the space, so that the most common CMOS chip can be used to read the hardware and obtain the distance of the generated space. For the human motion capture system based on inertial sensors, the initial signals include triaxial acceleration, triaxial angular velocity, and geomagnetic information [20]. By processing this information, the final motion characteristic parameters can be restored.

Data analysis is mainly used for the analysis of tactics in physical education teaching. The basic feature analysis software is used to analyze the captured moving targets and obtain the movement information such as displacement, velocity, angular velocity, and acceleration of the moving targets. Similarly, the technology also obtains two-dimensional and three-dimensional trajectory images, which provide accurate data for teaching.  Figure 1 shows the operation flow of the motion capture system.

## 4. Methodology

To explore the practicability and effectiveness of the basketball teaching and training resources, teaching design, media design, and virtual environment design incorporating motion capture technology, this study takes 50 students in the basketball elective class of normal university as experimental objects to carry out teaching experiments. After the test, the test results of all the subjects were balanced. All 50 students were divided into the experimental group and the control group. The final test results of the two groups were statistically analyzed using the *t*-test method, as shown in Table 1 and Figure 2.

From the outcomes shown in Table 2 and Figure 3, it can be seen from the basketball technology test results of the two groups of students that there is no significant difference in basketball technology between the two groups. Therefore, excluding the influence of proactive factors such as individual physical quality and basketball skill difference, the subjects meet the requirements of this experiment.

In this article, human bones are divided into hand bones and human bones, respectively. Hand bone joints are divided into 15 pieces and human bone joints are divided into 16 pieces. For each bone joint, the specific bone coordinate definition is shown in Figure 4.

According to the expression form of the rotation matrix, it can be found that the motion process of the carrier in space can be described by the form of the rotation matrix. This method can effectively avoid the problem of disordered joint motion orientation caused by different rotation sequences. Similarly, based on this principle, it is also applicable to the field of inertial motion capture, as shown in Figure 5.

When the image is placed in a three-dimensional space, there is the distance between any two points in the space, and the expression is given by the following equation:

(1) $$\begin{array}{c} S\left(t\right)=\frac{y\left(t\right)}{l}. \end{array}$$

The method maps the original data into a closed interval between 0 and 1 through linear transformation, as shown in (2), and achieves the function of scaling the original data signal equally.

(2) kj=RjDj×Uj×Rej.

The 0-mean normalization method processes the original data into a normal distribution set with a mean of 0 and a variance of 1, as shown in (3). However, this method is only applicable when the distribution form of the data is like the Gaussian distribution (statistical shape); otherwise, the result is not ideal.

(3) $$\begin{array}{c} R_{j}=\frac{f_{ij}}{Tj}\times S_{j}. \end{array}$$

Unit quaternion can be used to describe the rotation of a rigid body in a three-dimensional space. Its form is shown in (4), which is also a differential equation of quaternion.

(4) $$\begin{array}{c} S_{j}=\frac{1}{\sum_{i=1}^{n}\left(S_{r}\right)},\left(0<\left(S_{j}\right)\leq 1\right). \end{array}$$

Equation (4) represents quaternion, which is composed of angular velocity detected by gyroscope; its real part is 0, and *H*_*p*_ is the derivative of quaternion over time, as shown in the following equation:

(5) $$\begin{array}{c} D_{j}=\sum_{i=1}^{n}\left(H_{p}\times V_{p}\right). \end{array}$$

It is very important for this project to capture the user's actions and obtain the coordinates of joints in space. The system acquires real-time images through Kinect's color image camera, then converts the color images into HSV images by OpenCV, and binarizes them after the conversion is completed. According to the motion capture system, the power sequence, strength, and movement rhythm of the basketball players during the whole process of take-off, squats, and dribbles can be obtained. The system includes computer equipment, sensors, and data lines. Basketball players look back at their own motion images through computer equipment [21]. For long-term users, the database stores their training information. Based on this information, deficiencies in training can be found out, appropriate training methods can be recommended to users according to their personal situation, and the training effect of users can be recorded. When the picking robot works autonomously, its most important link is to locate the fruit target autonomously, which needs to rely on the robot's own powerful vision system. Hardware equipment mainly includes special near-infrared high-sensitivity camera, high-speed 3D motion data capture workstation, DIMS controller, and special cable. Furthermore, the software mainly includes high-precision 3D space calibration software, real-time high-precision 3D motion data capture software, data editing and format conversion software, and MotionBuilder 3D character animation software. Open GL in the above design only provides the modeling function of the basic geometric elements, which has certain limitations. The modeling of complex models can adopt 3ds Max, which is a powerful modeling tool. The 3ds Max can provide accurate modeling for complex 3D geometric entities, but unfortunately portability and rendering of objects are both insufficient in the 3ds Max program.

The “fixed-point shooting” teaching and training resources developed in this research and integrated with motion capture technology are used as experimental materials for teaching experiments. The experimental group uses teaching and training videos for teaching, while the control group adopts traditional teaching methods. The specific experimental arrangements are shown in Table 3.

After the experiment, the same test method was used to test the basketball skills of the two groups of students once again. The results and outcomes of comparing the technical level of the two groups of students before and after the experiment are shown in Table 4 and Figure 6 using paired sample *t*-test.

From Table 5 and Figure 7, it can be seen from the test results of the two groups of students before and after the experiment that there is a significant difference between the two groups of students in basketball technical level after the experiment. This observation shows that the basketball teaching and training resources designed to integrate action capture technology can improve students' learning efficiency of the basketball technology.

If we assume that *W* represents the state of the system at time *K*, *r*_*k*_ is the state of the system at the next time, and *r*_*i*_ is the process noise vector of the system and conforms to the expected characteristic of 0, then the state transition equation of the system can be obtained in the following form:

(6) $$\begin{array}{c} S\left(r_{k}\right)=\sum_{r_{k}\neq r_{i}}w\left(r_{i}\right)D_{r}\left(r_{k},r_{i}\right). \end{array}$$

Let *k* represent the measured value of the system at time *n*; *k* – 1 represents the process noise vector of the system and satisfies the characteristic that the expectation is 0. Then, the measurement equation can be expressed as shown in the following equation:

(7) $$\begin{array}{c} p_{n}^{k}=p_{n}^{k-1}+v_{n}^{k}. \end{array}$$

Among them, *p* represents the relationship between the system state and the system observation in the ideal state at time *k*, which realizes the transition from the system state to the observation state. For the noise covariance matrix of the system, since the process noise and the measurement noise are two uncorrelated signal forms, they satisfy the following equation:

(8) $$\begin{array}{c} B_{D}=\left|\log\left(\frac{I_{b}}{I_{f}}\right)\right|+D_{FB}. \end{array}$$

Therefore, the error covariance matrix associated with it is shown in the following equation:

(9) $$\begin{array}{c} \sigma =\sqrt{\mathrm{In}\left(1+\frac{v_{r}}{m^{2}}\right)}. \end{array}$$

With the prior estimation value *M*, the prior estimation of the system can be optimized through the measurement value *μ* of the system. Moreover, the measurement value and the prior estimation value of the noise system are fused in the following equation:

(10) $$\begin{array}{c} \mu =\mathrm{In}\left(\frac{m^{2}}{\sqrt{v_{r}+m^{2}}}\right). \end{array}$$

After obtaining the motion information of human joints, we must also use Cal3D software to render the bone motion; that is, after having different joints, we must also realize the 3D motion picture of the bone motion. A sensor node formed by combining a plurality of sensor devices can convert the action information in the process of completing the action into an electrical signal to upload, thereby realizing the requirements of subsequent logical operation, data storage, communication, and the like. In the motion capture system, there are certain errors and data noises in the human motion characteristic data collected by inertial sensors, which need to be filtered and corrected. Since the triaxial accelerometer has good static characteristics and there is no accumulated time error, the attitude angle calculated by the triaxial accelerometer can be used to correct the roll angle and pitch angle calculated by the gyroscope. Pose software is used to build a three-dimensional model of a basketball player's body, including effective fixation of specific functions such as bone structure and some joints, and filter noise in the information. The main function of the data conversion is to convert different types of data into the same data that can be used uniformly. At the same time, in data processing, the characteristic parameters of human motion need to be solved at a high speed. According to the relevant fusion algorithm, the effective motion characteristics and trajectories are analyzed from the original signals. These characteristic parameters are combined with the 3D motion model to drive the model and to simulate the real human motion in real time.

After the experiment, all the scores of basketball skills of the two groups of students were compared and counted in detail (see Table 6 and Figure 8). Among them, the experimental group had more than 80 points, and a total of 5 students were rated as excellent, with an excellent rate of about 24%; the control group's excellent rate was about 11%. The failure rate was 15.17% in the experimental group and 35.23% in the control group. The pass rate of the experimental group was about 80.63%, while that of the control group was 67.73%.

In the motion capture system, the restoration effect of the motion is the standard to evaluate the advantages and disadvantages of the motion capture products. In the system designed in this paper, referring to human kinematics and anatomy principles, a motion capture platform based on 3D perspective of bone stack is built through relevant software. According to the action extraction technology of the basketball real-time video, the important target features can be extracted, and the robot can finally realize autonomous important positioning and autonomous operation. At the same time, it can edit, delete, interpolate, and filter the three-dimensional spatial position information of the target at any time point in the captured three-dimensional motion data, and the modified complete data can be converted into the general motion data format of CSM/BVH/TRC/FBX and other 3D and CG software. The capture based on human body is to first separate the image of the human body from the depth map, and then, through the evaluation and identification of pixels, match it with the human body model existing in the system, to obtain the model conforming to the height and bone type. This belongs to the control problem of the model. The designer inputs the orientation and target position of the manipulator end. The trajectory planning of the system is mainly responsible for determining the motion, shape, speed, and time of the joint trajectory reaching the target. According to the requirements of the practical application, it is difficult for a single sensor module to meet the working requirements. The information needed in human posture recognition is complex and diverse, including physical and physiological information such as acceleration, angular velocity, or heart rate. Then, it is sent to the upper computer of PC through wireless transmission. After analyzing the signals, the upper computer is used to drive the three-dimensional motion model in real time. It should be noted that the three-dimensional motion model can be constructed through structural modeling of limbs.

## 5. Result Analysis

This system is developed based on IOS platform and Windows platform. Because Kinect and the nine-axis inertial sensor are developing simultaneously, the data obtained are more accurate. Motion capture technology is to track the motion trajectories of nodes with key information in some virtual simulation results of some organisms in a fixed time domain and convert the motion trajectories of key points into 3D motion processes that can be mathematically expressed and combined. The system needs to have the function of motion simulation. It can be virtualized and modeled in combination with the actual scene to make it a virtual scene like the real environment and perform 3D simulation on the characters in the scene. The main goal of the edge detection algorithm is to detect the maximum value of the gradient change and to suppress noise by optimizing the gradient value to effectively find the position of the edge. The modified complete data can be analyzed through a specific data analysis system for position information, motion speed, angle, angular velocity, acceleration, etc. of the moving target point, and the corresponding data chart can also be compared and displayed by two sets of data. The system gives the athlete's initial position, target position, and several key points through which the path between them passes. In this case, appropriate trajectories are designed to perfect the parts not given in the athlete's trajectory. It can be converted into characteristic parameters that can be used to drive the movement of the human body model, thus realizing real-time and accurate tracking of the real human body movement by the model. At the same time, the upper computer can also display and store the movement characteristic data in real time, thus realizing comprehensive online and real-time supervision.

In general, in human motion capture, the range of bone motion must be biomechanically limited to make it move within a reliable range.  Table 7 defines the types of human and hand joints and their range of motion, respectively.

To capture human body posture using inertial motion sensors and realize the capture of the human body movement posture, according to the tree structure of human body introduced above, the hierarchical modeling method is adopted in this paper. The whole human body is regarded as a skeleton tree composed of rigid bodies. In the skeleton tree, except the designated root node, each bone is connected by hinges, the bones are divided into parent-child relationships, and the child nodes move around the parent node.  Figure 9 depicts the basic skeleton tree structure of the human body.

Human motion capture based on inertial sensing regards human body as a tree structure composed of multiple rigid bodies. To accurately capture human motion, sensor nodes need to be fixed at each calibration position, which is the basic link to realize motion capture. The software and hardware products are combined to measure the joint angles of the two arms through four nine-axis inertial sensors, to track the motion track and motion state of the whole arm. Before the data collection, the exact location of the sensor installation and the corresponding location between the sensor and the human body should be confirmed. In addition, the human body cannot contain any metal products, which will interfere with the magnetic field and affect the collection of human body data. From the actual situation, motion capture is mainly to eliminate the influence of the background, take the individual athlete as the capture object, and transmit the captured video to the system for comprehensive processing. On this basis, the corresponding human body model can be obtained, and the corresponding capture result can be obtained after parameterization processing of the human body model in the system. In the process of real-time sensor acquisition, due to the fast speed of basketball movement, there will inevitably be more noise, which can be minimized through filtering methods. Motion capture is an important part of the system work, which refers to the process that the system captures and outputs the motion track of the marker ball in the key part of the moving target in the designated space through 8 near-infrared high-sensitivity cameras. Through these devices, the motion status of the moving objects is captured, and the captured information is recorded in the form of images and further processed on the computer, to obtain the spatial coordinates of different athlete models.

To apply the extended Kalman filter technology to the actual scene of nonlinear changes, firstly, a differential equation group of nonlinear changes needs to be defined, as shown in the following equation:

(11) $$\begin{array}{c} M_{k}=c_{k}^{d}M_{k-1}. \end{array}$$

The process noise matrix *k* is composed of a set of process noise vectors *r*_*i*_, as shown in the following equation:

(12) $$\begin{array}{c} T_{r}=\frac{1}{N}\sum_{i=i_{0}}^{k}r_{i}r_{i}^{T}. \end{array}$$

In addition, the measurement function is a nonlinear state equation as follows:

(13) $$\begin{array}{c} \text{PR}\left(k\right)=T_{r}\left(k\right)-V_{r}\left(k\right), \end{array}$$

where function *S*_*N*_ is the observation equation of the system and *n* is the measurement error vector expected to be 0 and is represented by measurement noise matrix *N*_0_, as illustrated in the following equation:

(14) $$\begin{array}{c} S_{N}\left(k\right)=\frac{\left|\Delta N/N_{0}\right|}{\left|\Delta k\right|/\left(k_{\max}-k_{\min}\right)}. \end{array}$$

Next, the data of heterogeneous sensors need to be modeled and analyzed. Our goal is to obtain the rotation matrix between the sensor coordinate system and the global world coordinate system by processing the motion data collected by the sensors. Therefore, it is first necessary to use sensors to collect initial human motion characteristic signals and obtain vector data of each sensor according to its vector representation.  Table 8 and Figure 10 show the dynamic measurements of gyroscopes and magnetometers, respectively.

## 6. Discussion of the Findings

In the system designed in this paper, sensors are deployed at the key nodes of the human body, and the motion information of the key nodes is captured by the sensors; thus, the motion situation of the whole human body can be calculated. How to choose the location of key nodes is a key link and question. In the process of using Kinect as data acquisition, Kinect usually acquires 17 different joint points. However, during the acquisition process, due to the acceleration of human body movement, the problem of blocking images of some joints due to human body movement will occur. Compared with sensor nodes, the wearing position of the mobile equipment is not fixed, which will affect the recognition results of the system. When detecting motion information through sensors, the equipment can be placed in a fixed position to avoid this or other similar effects. The movement track of the key bones is placed on the constructed virtual characters, and the training process of the virtual athletes is controlled by controlling the movement track of the key bones. This method is convenient for mastering the technical characteristics of the basketball athletes. In the actual training process, the system can digitize the athletes' movement process and various parameters; in particular, the parameter processing of various details can effectively improve the athletes' technical level. It can also monitor various physical skill parameters of athletes in real time, such as heart rate, blood pressure, and cardiopulmonary function. To capture the human posture accurately, we must have an accurate grasp of the human skeleton structure and its movement state. Therefore, in the process of analyzing the human body structure, it is necessary to reasonably divide the human body structure and extract the key bone movement characteristics in the process of human body movement to facilitate understanding.

The promotion process of the basketball skills by athletes through virtual simulation technology needs the support of mathematical statistics function. Therefore, the system needs to have mathematical statistics function, which can be combined with the system for comprehensive analysis in actual analysis. Of course, besides analyzing the structure of the model, we also need to define the motion angles of each bone structure. In real life, we can find that, due to the limitations of bone structure and so on, the motion angles of many joints are limited in scope and cannot move 360 degrees in all directions. Using the principle of gradient algorithm, by changing the gradient of the image, the partially blurred part of the image is made clear to find the obvious edge of the image. Data processing includes full-automatic 3D data reconstruction and automatic tracking of identification points. Operators can reconstruct and track motion capture data automatically and manually to obtain accurate 3D data.

The sensor is installed on the athlete's simulation model. The sensor belongs to a particular tracking device. It can track the athlete to determine its position and to control the motion trajectory. The fineness of the motion capture can be measured by the number of sensors. The aim of the physical education teaching system is to correct students' teaching actions. In this paper, combined with the practice of physical education, the application of this system is only suitable for the training in relatively specialized disciplines in colleges and universities, such as basketball and golf courses. After the adoption of this system, the number of free-hand gymnastics, ball gymnastics, and tumbling exercises of athletes has been significantly increased. Moreover, the flexibility of the athletes has been greatly improved, which is conducive to reducing the probability of collision injuries of the athletes.

## 7. Conclusions and Future Work

This paper constructs a virtual simulation system for students' sports training. The experimental results show that the system can promote the physical training of the basketball players and can significantly improve the running speed, body flexibility, and jumping capability of the basketball players. The Kinect color camera and depth camera are used to obtain the shooting arm data of the user, and four nine-axis inertial sensors are used to complete the measurement of the joint angles of the two arms to obtain a large amount of data. Combined with the existing motion capture technology, based on current optical and mechanical motion capture, the existing research theory of motion capture technology is analyzed and summarized. In addition, a real-time capture method of human posture based on inertial sensing is proposed. Combined with relevant research ideas, the design content and scheme are summarized and analyzed, and the overall design scheme and technical route are proposed. The system uses personalized recommendation algorithms such as data processing algorithms, and each part of the system is constructed through distributed structure. Under the joint action of each part, the system can effectively analyze the user's needs and solve the user's actual needs. Through testing, it is concluded that the system constructed in this study has significant reliability and effectiveness. In the future, we will consider more experimentation and larger datasets, along with several other parameters, to study the generalization and validation of the proposed idea. Similarly, other motion capture methods should be investigated to support the findings and outcomes of our research.

## Figures and Tables

**Figure 1:** Operation flow of motion capture system.

**Figure 2:** Personal physical fitness test results.

**Figure 3:** Results of basketball technical test.

**Figure 4:** Definition of human body skeleton coordinates.

**Figure 5:** Definition of Euler angle.

**Figure 6:** Paired sample statistics.

**Figure 7:** Paired sample test.

**Figure 8:** Comparison of basketball skill scores.

**Figure 9:** Bone tree structure.

**Figure 10:** Dynamic measurements of gyroscopes and magnetometers.

**Table 1:** Personal physical fitness test results.

Grouping	Mean value	Standard deviation
Experimental group	4.63	0.58
Control group	5.89	0.77

**Table 2:** Results of basketball technical test.

Grouping	Mean value	Standard deviation
Experimental group	36.33	10.24
Control group	40.15	9.83

**Table 3:** Experimental arrangement.

Experimental arrangement	Student behavior	Teacher behavior	Observer behavior
Grouping	Organizing and testing personal physical fitness and basketball skill tests	Organizing tests and determining grouping	Recording all the test indexes of the students and cooperating with the teachers to determine the grouping
Teaching evaluation	Basketball technical test	Organization test	Recording test results

**Table 4:** Paired sample statistics.

	Mean value	Standard deviation
Pretest of experimental group	35.39	9.85
Posttest of experimental group	60.97	12.22

**Table 5:** Paired sample test.

	Mean value	Standard deviation
Pretest of experimental group	4.88	5.51
Posttest of experimental group	9.12	8.92

**Table 6:** Comparison of basketball skill scores.

Group	Rate of excellence (%)	Pass rate (%)	Failure rate (%)
Experimental group	24	80.63	15.17
Control group	11	67.73	35.23

**Table 7:** Description of human joints.

Joint name	Parent bone	Joint type	Variance	Limit of range of activities (degree)
Vertebra	No	—	—	0–50
Cervical vertebra	Thoracic bone	Universal joint	2	0–70
Shoulder joint	Thoracic bone	Universal joint	2	0–180
Elbow joint	Upper arm skeleton	Hinge	1	0–145

**Table 8:** Dynamic measurements of gyroscopes and magnetometers.

	Sampling points	Initial acceleration (g/LSB)
Gyroscope	45.36	98.02
Magnetometer	69.63	120.33

## Data Availability

The data used to support the findings of this study are included within the article.
